# Positive Direct Immunofluorescence in Rowell Syndrome: Further Support for a Subtype of Cutaneous Lupus Erythematosus

**DOI:** 10.7759/cureus.85097

**Published:** 2025-05-30

**Authors:** Ashley Bissenas, Mitchell Bourne, Arthur M Samia, Kiran Motaparthi

**Affiliations:** 1 Department of Dermatology, University of Florida College of Medicine, Gainesville, USA; 2 Department of Internal Medicine, University of Florida College of Medicine, Gainesville, USA

**Keywords:** diagnostic criteria, direct immunofluorescence, erythema multiforme, lupus erythematosus, rowell syndrome

## Abstract

Rowell syndrome (RS) is a rare clinical entity characterized by erythema multiforme (EM)-like lesions and lupus erythematosus (LE). Immunologic findings associated with RS include a speckled antinuclear antibody (ANA) pattern, positive rheumatoid factor (RF), and anti-Ro (SS-A)/anti-La (SS-B) antibodies. While direct immunofluorescence (DIF) positivity is a hallmark of cutaneous LE (CLE), recent diagnostic criteria for RS suggest DIF should be negative, raising debate over whether RS is a distinct disease or a CLE variant.

We present the case of a 42-year-old woman with systemic lupus erythematosus (SLE) who developed a diffuse, blistering rash consistent with RS. DIF of lesional skin demonstrated immunoreactivity for IgG, complement C3, and IgM along the basement membrane zone, contradicting the proposed RS criteria.

This case reinforces the argument that RS is best classified as a CLE subtype rather than a distinct disease. The patient’s clinical, serologic, and histopathologic findings, including DIF positivity, support this classification.

## Introduction

Rowell syndrome (RS) is characterized by erythema multiforme (EM)-like lesions with serologic and immunologic evidence of lupus erythematosus (LE) [1]. Immunologic findings supportive of RS include a speckled pattern of antinuclear antibodies (ANAs), positive rheumatoid factor (RF), and the presence of anti-Ro (SS-A)/anti-La (SS-B) antibodies [2]. Lesional direct immunofluorescence (DIF) is another method described in the differentiation of RS from other diseases [3]. Controversy still remains as to whether RS is a distinct entity or a subtype of LE. The major types of LE include systemic and cutaneous, with the subacute and chronic forms most commonly associated with RS [1,4]. The most recent diagnostic criteria posit that DIF should be negative in RS [1]. Herein, we present a patient diagnosed with RS and positive DF typical of LE, adding support to the inclusion of RS as a subtype of CLE.

## Case presentation

A 42-year-old woman presented to the emergency department for a diffuse, blistering rash over her arms, legs, chest, abdomen, and back of five days duration. One week prior to hospitalization, she presented to an urgent care facility for suspected acute otitis media and was prescribed cephalexin. The patient noted that a rash appeared two days after starting the antibiotic, and it originally started on her arms and abdomen, which she described as painful. She was previously treated with hydroxychloroquine and azathioprine and is currently on mycophenolate mofetil 250 mg twice daily for her SLE. The patient’s past medical history also included stage IV chronic kidney disease (CKD) secondary to lupus nephritis, non-insulin-dependent diabetes mellitus, and hypertension. Vitals were hemodynamically stable (Table 1). On physical exam, there were dusky targetoid plaques with overlying bullae and erosions, as well as annular hyperpigmented macules and patches varying from 2 to 5 cm in size (Figures 1-3). The distribution included the extremities, trunk, and face; however, the conjunctiva and genitalia were spared. An ulcer was also noted on the inferior lip (Figure 2). The patient denied pain or pruritus. The initial differential diagnosis was generalized bullous fixed drug eruption secondary to cephalexin versus RS. Biopsies for routine histopathology and DIF were performed. Histopathology demonstrated epidermal necrosis overlying a re-epithelializing epidermis, interface dermatitis, and perivascular and periadnexal lymphocytic infiltrate without eosinophils (Figures 4, 5). Of note, the DIF of lesional skin demonstrated immunoreactivity for IgG, complement C3, and IgM in a granular pattern along the basement membrane zone. Laboratory evaluation demonstrated ANA with speckled pattern, elevated double-stranded DNA antibody, elevated SS-A 60 (anti-Ro60) antibody, equivocal SS-A 52 (+anti-Ro52) antibody, equivocal SS-B (anti-La) antibody, and normal RF (Table 2). The patient was diagnosed with RS, and the dose of mycophenolate mofetil was increased to 500 mg twice daily, hydroxychloroquine 200 mg daily was started, and given the extent of her disease, prednisone 40 mg daily was also started with close blood glucose monitoring given her uncontrolled diabetes. The subsequent plan for this patient was to start anifrolumab in the outpatient setting for her SLE and RS; however, the patient developed necrotizing fasciitis of her right upper extremity 11 days after her admission. At this point, prednisone was discontinued as it was no longer a suitable option given her critical state. Intravenous immunoglobulin was started during continuous renal replacement therapy at 30 mg/kg/hour, increasing to a rate of 120 mg/kg/hour until 35 g total was delivered. She underwent debridement surgeries for her necrotizing fasciitis and was eventually stabilized. At the one-month follow-up, the patient had no new lesions, and prior lesions had healed with dyspigmentation and scarring, which can occur in subacute CLE and RS (Figure 6). 

**Table 1:** Vital signs

	Reference range	Patient’s value
Blood pressure (mmHg)	90-120/60-80	149/78
Temperature (℉)	97.0-98.9	97.8
Heart rate (beats per minute)	50-90	89
Respiratory rate (breaths per minute)	12-20	18
SpO_2_	95%-100%	99%

**Figure 1:** Dusky patches, some with overlying bullae, on the eyelids Note: Written informed consent to include these images in an open-access article was obtained from the patient.

**Figure 2:** Dusky patches, some with overlying bullae, on the periocular skin; an ulcer on the inferior lip was noted Note: Written informed consent to include these images in an open-access article was obtained from the patient.

**Figure 3:** Abdomen and groin with annular dusky patches, some with overlying bullae Note: Written informed consent to include these images in an open-access article was obtained from the patient.

**Figure 4:** Lesional biopsy demonstrating epidermal necrosis overlying a re-epithelializing epidermis and a cell-poor interface dermatitis, perivascular and periadnexal lymphocytic infiltrate. Deep melanophages and eosinophils were absent

**Figure 5:** Lesional biopsy demonstrating epidermal necrosis overlying a re-epithelializing epidermis with degeneration of basal cells (H&E, 20x magnification)

**Table 2:** Autoimmune antibody results

	Negative value	Positive value	Patient’s value
ANA antibody titer	<1:40	>1:80	1:1280
Double-stranded DNA antibody (IU/mL)	<4	>10	87
SS-A 60 antibody (AU/mL)	<29	>41	41
SS-A 52 antibody (AU/mL)	<29	>41	33
SS-B antibody (AU/mL)	<29	>41	36
Rheumatoid factor (IU/ML)	<14	>14	<10.0

**Figure 6:** Abdomen and groin at one-month follow-up, with residual scarring and dyspigmentation Note: Written informed consent to include these images in an open-access article was obtained from the patient.

## Discussion

RS is a disease characterized by both LE and EM-like lesions, described as pruritic, annular, erythematous, red or violet plaques with blisters, often found on the limbs, face, chest, and mouth [5]. The disease primarily affects women in an 8:1 ratio [6]. Studies vary as to whether the most commonly affected age group is middle-aged or elderly women [6,7]. The exact etiology of RS is unknown. However, it has been linked to estrogen, toll-like receptors, certain drugs, and sun exposure [8-10].

Similarly, CLE predominantly affects women in a 3:1 ratio [11]. The most common age range affected is the young to middle-aged [11]. The pathogenesis of CLE is multifactorial, including UV radiation and autoimmune dysregulation [12]. Subtypes of CLE include acute, subacute, and chronic. 

The diagnostic criteria for RS have varied over the years and were initially described in 1963 by Rowell [13]. The most recent criteria proposed by Torchia et al. [1] states that all four major and one minor criteria must be present for diagnosis. The major criteria include the presence of chronic cutaneous lupus erythematosus; EM-like lesions; at least one positivity among speckled ANA, anti-Ro/SSA, and anti-La/SSB antibodies; and negative DIF of EM-like lesions [1]. 

Although there are no specific criteria for the diagnosis of CLE, serological findings often include positive ANA, anti-Ro/SSA, and dsDNA [14]. Additionally, CLE is classically characterized by DIF positivity, causing some to posit that RS is a distinct disease [15]. However, many experts now agree that RS is a variant of CLE [3,5]. DIF can appear negative due to the degradation of the immune reactants [16]. This may be due to the fact that epidermal necrosis, which accounts for the dusky appearance of EM-like lesions in RS, can result in a false-negative DIF [17]. Thus, we posit that DIF negativity should be removed from the diagnostic criteria for RS, as DIF supports the classification of RS as a subtype of CLE (Table 3).

**Table 3:** Proposed differences in RS classification, as a subtype of CLE RS: Rowell syndrome, CLE: cutaneous lupus erythematosus.

	Torchia et al. (2012) [1]	Proposed differences
Direct immunofluorescence findings	Negative DIF on lesional EM-like lesions	Positive or negative DIF on lesional EM-like lesions
Autoantibody findings	At least one positivity among speckled ANA, anti-Ro/SSA, and anti-La/SSB antibodies	At least one positivity among speckled ANA, anti-Ro/SSA, and dsDNA antibodies

The patient’s periocular involvement and annular lesions, which are classic for subacute CLE, and the ulcer on her inferior lip, which likely reflected her SLE, are additional clinical evidence that RS may be a variant of CLE [18]. Additionally, while uncommon, scarring and ulceration can occur in severe CLE, as in this case [18]. Although RS dermatological findings have been described as EM-like, several cases of LE with EM-like lesions have been documented. [1] Moreover, while both RS and LE are associated with autoimmune mechanisms, EM is associated with infections and medications. [19] While other published cases of RS have continued to uphold DIF negativity for diagnosis, the case presented provides further support that RS is a variant of CLE, as it is clinically, pathologically, and serologically indistinguishable.

## Conclusions

RS remains a debated topic in dermatology, with ongoing discussion about whether it represents a distinct disease or a variant of cutaneous lupus erythematosus. The case presented reinforces the latter classification, with prior case reports similarly upholding this classification. The patient's physical exam findings of dusky, targetoid plaques, and bullae and serological results of positive ANA, dsDNA, and SS-A antibodies were consistent with RS. However, the positive direct immunofluorescence is more consistent with a diagnosis of CLE. While current diagnostic criteria for RS include DIF negativity, this case report highlights how DIF may be positive. This may, in part, be due to the potential for false-negative DIF due to immune reactant degradation or epidermal necrosis. Thus, this case report implies the need for reclassification of RS to a subtype of CLE, rather than a separate entity.
